The article "Comparison between the Severity Scoring Systems A-DROP and CURB-65 for Predicting Safe Discharge from the Emergency Department in Patients with Community-Acquired Pneumonia" was published in 2022. Journal: Emerg Med Int.

# Comparison between the Severity Scoring Systems A-DROP and CURB-65 for Predicting Safe Discharge from the Emergency Department in Patients with Community-Acquired Pneumonia

**DOI:** 10.1155/2022/6391141

**Published:** 2022-04-18

**Authors:** Thanya Limapichat, Suvanun Supavajana

**Affiliations:** Department of Emergency Medicine, Songklanagarind Hospital, Faculty of Medicine, Prince of Songkla University, Songkhla, Thailand

## Abstract

**Background:**

In most community-acquired pneumonia (CAP) treatment guidelines, the Pneumonia Severity Index (PSI) and CURB-65 are used as prognostic tools. Recently, simpler and more effective predictive tools for CAP treatment, such as the A-DROP scoring system, have been developed. However, no study has performed a comparative evaluation to identify the superior tool for predicting when patients can be discharged safely.

**Objectives:**

To compare the performances of A-DROP and CURB-65, simple predictive tools for CAP, based on 30-day death rates and 72-hour revisit rates for CAP following discharge from the emergency department (ED).

**Method:**

This single-center retrospective observational study enrolled patients who were at least 18 years old and diagnosed with CAP at the Songklanagarind Hospital ED from January 2015 to April 2021. Following a severity assessment using the A-DROP and CURB-65 scoring systems, the 30-day mortality rates and 72-hour revisit rates after discharge from the ED were compared.

**Results:**

A total of 408 patients were enrolled in this study. Six (1.47%) died within 30 days after presentation, whereas 29 (7.1%) returned to the ED within 72 hours after discharge. Most patients (72%) who revisited the ED were over the age of 65 years. The areas under the receiver operating characteristic curves for the prediction of 30-day mortality were 0.756 (95% confidence interval [CI]: 0.526–0.987) and 0.808 (95% CI: 0.647–0.970) for A-DROP and CURB-65, respectively. The areas under the receiver operating characteristic curves for the prediction of 72-hour revisit were 0.617 (95% confidence interval [CI]: 0.507–0.728) and 0.639 (95% CI: 0.536–0.743) for A-DROP and CURB-65, respectively.

**Conclusion:**

A-DROP and CURB-65 yield similar results and can be used to assess low-risk patients with CAP for discharge from the ED. Older patients, even those with low-risk scores, should be particularly considered for admission to a short-term observation unit or ward.

## 1. Introduction

Pneumonia is an infectious disease that causes inflammation of the air sacs in the lungs. In Thailand, pneumonia is the third most prevalent infectious disease [1]. In the United States, more than 1.5 million people with pneumonia are admitted to hospitals every year [2]. Furthermore, according to several studies, community-acquired pneumonia (CAP) accounts for approximately 3 million cases and 1.6 million hospitalizations per year in the United States [3, 4]. In addition, in Italy, it is reported to be the most prevalent reason for hospitalization and the leading cause of death [5].

The article "Comparison between the Severity Scoring Systems A-DROP and CURB-65 for Predicting Safe Discharge from the Emergency Department in Patients with Community-Acquired Pneumonia" was published in 2022. Journal: Emerg Med Int.

The total number of patients with CAP admitted to Songklanagarind Hospital's emergency department (ED) in 2019 was 1,104. Among them, 657 were men, and the majority were under the age of 65; 207 patients were allowed to return home. Ten patients (4.8%) returned to the ED for treatment [6]. Patients returning to the ED with symptoms that have either not improved or have worsened is an ongoing issue for emergency care physicians. The phenomenon of patients returning to the ED for retreatment is critical from the standpoint of the healthcare system; it leads to greater congestion in the ED as well as higher healthcare expenses [7].

For patients with CAP, in addition to appropriate management of this condition, prognosis tools are utilized to determine whether patients should be treated as outpatients or inpatients [8], since all those with pneumonia do not require hospitalization [5]. The Pneumonia Severity Index (PSI) and CURB-65 are used as predictive tools in most CAP treatment guidelines, although the PSI score is not currently adequate for use in the ED for outpatient treatment. The PSI score consists of 20 components, and not all of them are assessed in all patients, especially in those presenting with mild symptoms and undergoing outpatient treatment.

Many studies have developed new prognostic tools for CAP [9–12]. The A-DROP score was introduced by the Japanese Respiratory Society in 2006 [11]. It proposes a 6-point scale (0–5) to assess the clinical severity of CAP and consists of five parameters: (1) age (male ≥70 years and female ≥75 years); (2) dehydration (blood urea nitrogen [BUN] ≥ 21 mg/dL); (3) respiratory failure (SaO_2_ ≤ 90% or PaO_2_ ≤ 60 mmHg); (4) orientation disruption (confusion); and (5) low blood pressure (systolic blood pressure ≤90 mmHg). A-DROP is as an adaptation of the CURB-65, which was published by the British Thoracic Society in 2002 and includes the parameters of confusion, BUN > 7 mmol/L (20 mg/dL), respiratory rate ≥30/min, low blood pressure (diastolic ≤60 mmHg or systolic <90 mm Hg), and age ≥65 years [12]. Both are simple, reliable, and widely used tools for assessing patients with CAP. Patients are stratified into low, intermediate, and high-risk groups, among which the low-risk group is scored 0–1 in both scoring systems and can be treated as outpatients [11, 12].

The article "Comparison between the Severity Scoring Systems A-DROP and CURB-65 for Predicting Safe Discharge from the Emergency Department in Patients with Community-Acquired Pneumonia" was published in 2022. Journal: Emerg Med Int.

To the best of our knowledge, there is no comparative study of the efficacy of these tools to predict which patients with CAP can be safely discharged from the ED. In addition, there are no clear clinical practice guidelines for the disposition of patients with CAP from the Songklanagarind Hospital ED. As a result, physicians at the Songklanagarind Hospital use the CURB-65, A-DROP, and/or PSI as well as their personal experience to make treatment decisions, which leads to great variability in clinical practice related to the management of this group of patients at our department. We believe that identifying the most effective and safest tool for the discharge of patients with CAP will benefit both the patients and medical personnel. This would lead to the tool being utilized in the standard management of all patients with CAP, and consequently, to lower death and hospital revisit rates. This study aimed to compare A-DROP and CURB-65 because these are the easiest and quickest tools to use.

## 2. Patients and Methods

### 2.1. Study Design and Setting

This single-center, retrospective, observational study included patients who were at least 18 years old and diagnosed with CAP at the ED of Songklanagarind Hospital, a tertiary referral and academic hospital at the Hat Yai Campus of Prince of Songkla University in Southern Thailand. Approximately 50,000 patients visit the ED of this hospital each year. Patient data from January 2015 to April 2021 were retrieved from the hospital's electronic medical record database. The Research Ethics Committee of the Faculty of Medicine, Prince of Songkla University approved the study (REC 63-355-20-4). Patient consent was not required because data anonymity was maintained, and standard treatment was provided for all patients. All research data were encrypted; only the researchers had access to the data.

### 2.2. Study Population

In this study, CAP was defined as pneumonia in a patient who contracted an infection outside the hospital and who was not hospitalized or in a care center for more than 14 days prior to presentation [13]. Pneumonia was defined as the presence of a new radiographic infiltrate and at least one of the following criteria: fever (≥38°C) or hypothermia (<35°C), new cough with or without sputum production, pleuritic chest pain, dyspnea, and altered breath sounds on auscultation [14]. This study excluded patients with hospital-acquired pneumonia (HAP), active thoracic malignancy (primary lung cancer and/or lung metastasis), immunosuppression due to neutropenia after chemotherapy, HIV infection, solid organ transplantation, corticosteroid or other immunosuppressive agent therapy (including maintenance corticosteroid therapy at any dose and chemotherapy), pulmonary embolism, active pulmonary tuberculosis, complicated pneumonia or multiple underlying diseases, no caregiver, COVID-19 pneumonia as well as those who were nursing home residents, had incomplete medical records, refused hospitalization, and died from a cause other than pneumonia within 30 days after discharge.

The article "Comparison between the Severity Scoring Systems A-DROP and CURB-65 for Predicting Safe Discharge from the Emergency Department in Patients with Community-Acquired Pneumonia" was published in 2022. Journal: Emerg Med Int.

The sample size of the study was calculated based on the study by Shindo et al. [15], using the one proportion formula and the N4Studies program [16, 17]. To compensate for the expected dropout rate, 10% of the sample size was added, resulting in a total sample size of 408 patients. The number of patients was calculated using the following formula to estimate the infinite population proportion:

(1) $$\begin{array}{c} n=\frac{z_{1-\left(\alpha /2\right)}^{2}\;p\left(1-p\right)}{d^{2}}, \end{array}$$

where estimated mortality rate *p*=0.095 [15], error d = 0.03, *α* = 0.05, *Z* (0.975) = 1.96, sample size (*n*) = 367, and 10% incomplete data = 408.

### 2.3. Data Collection

The data obtained from the electronic medical records included the patient sex, age, comorbidities (i.e., neoplastic disease, chronic lung disease, congestive heart failure, chronic renal disease, chronic liver disease, central nervous system [CNS] disorder, and diabetes), clinical parameters (i.e., orientation disturbance (confusion), systolic blood pressure <90 mmHg or diastolic blood pressure ≤60 mmHg, pulse rate ≥125/min, respiratory rate ≥30/min, SaO_2_ ≤ 90% (or PaO_2_ ≤ 60 mmHg)), laboratory findings (BUN > 20 mg/dL for CURB-65 and ≥21 mg/dL for A-DROP), radiographic findings (bilateral lung involvement ≥ two zones involved), use of antibiotics within the previous 90 days, and outcome measures (i.e., recovery, revisit within 72 hours, and 30-day mortality).

### 2.4. Outcome Measures

The primary outcomes were the 30-day mortality and 72-hour hospital revisit rates in patients with CAP discharged based on the A-DROP and CURB-65 assessment scores. The goal of the study was to identify a simple score that allows safe discharge of patients with CAP from the ED. The secondary outcome was the characteristics of the revisit group.

### 2.5. Statistical Analysis

All data were analyzed using the R software version 4.1.1. Descriptive statistics, that is, the frequency, percentage, mean and standard deviation, or median and range, were employed to present the demographic and clinical variables, outcome measures, 30-day mortality, and rate of hospital revisit within 72 hours in patients discharged from the ED based on the A-DROP and CURB-65 scoring systems. The areas under the receiver operating characteristic (ROC) curves (AUCs) for predicting 30-day mortality and hospital revisit within 72 hours between the A-DROP and CURB-65 scoring systems were compared. The significance of the *p*-value was set at 0.05.

The article "Comparison between the Severity Scoring Systems A-DROP and CURB-65 for Predicting Safe Discharge from the Emergency Department in Patients with Community-Acquired Pneumonia" was published in 2022. Journal: Emerg Med Int.

## 3. Results

A total of 639 patients with pneumonia were discharged from our ED during the study period. Of them, 85 patients were excluded; among which 43 had an active thoracic malignancy, 17 had immunosuppression, 15 contracted HAP, 8 had active pulmonary tuberculosis, and 2 died from a cause other than pneumonia within 30 days after presentation. Thus, 554 patients with CAP were discharged from the ED. Of those, 144 patients had incomplete data, and another 2 refused to be hospitalized. Hence, a total of 408 patients were included in this study (Figure 1).

The baseline characteristics and outcome measures for our study patients are shown in Table 1. The median age was 67.9 years (interquartile range, 58–81). Six (1.47%) of the 408 patients died within 30 days after presentation, whereas 29 (7.1%) returned to the ED within 72 hours after discharge. Four (13.7%) of the 29 patients who returned within 72 hours died within the following 30 days. The 30-day mortality data and the 72-hour revisit rates with respect to the severity scores calculated using A-DROP and CURB-65 are shown in Table 2. The distribution of the revisit group based on A-DROP and CURB-65 scores is shown in Table 3. The most frequent rates were as follows: age ≥65 years (72.4%), respiratory rate ≥30 breaths per minute (48.3%), and BUN >20 mg/dL (34.5%).

The ROC curves for the 30-day mortality based on the two scoring methods are shown in Figure 2. The ROC analysis for the prediction of 30-day mortality yielded AUCs of 0.756 (95% confidence interval [CI]: 0.526–0.987) and 0.808 (95% CI: 0.647–0.970) for A-DROP and CURB-65, respectively. The ROC curves for the 72-hour revisit are shown in Figure 3. The ROC analysis for the prediction of hospital revisit rate within 72 hours yielded AUCs of 0.617 (95% confidence interval [CI]: 0.507–0.728) and 0.639 (95% CI: 0.536–0.743) for A-DROP and CURB-65, respectively. There was no statistically significant difference in the AUCs between A-DROP and CURB-65. Meanwhile, a significant increase in mortality was observed in patients with higher CURB-65 and A-DROP scores.

There were 153 patients in the non-low-risk group (A-DROP and/or CURB-65 score ≥2) who were discharged from the ED; only 63 (41%) had a documented severity score, and the remaining 90 (59%) were discharged without a determined score. Three (3.3%) of the 90 patients discharged without either an A-DROP or CURB-65 CAP severity score died within 30 days and another 9 (10%) revisited the ED. No patient with an A-DROP or CURB-65 score of 5 was discharged because they were considered high risk according to both scoring systems.

The article "Comparison between the Severity Scoring Systems A-DROP and CURB-65 for Predicting Safe Discharge from the Emergency Department in Patients with Community-Acquired Pneumonia" was published in 2022. Journal: Emerg Med Int.

## 4. Discussion

The purpose of our study was to evaluate whether A-DROP and CURB-65 could be used to safely discharge patients with CAP from the ED based on 30-day mortality rates and 72-hour revisit rates. Our findings indicated that the A-DROP scoring system yielded equivalent results to those of the CURB-65 assessment tool. Similar to our investigation, a retrospective study by Shindo et al. published in 2008 compared the efficacy of A-DROP and CURB-65 in assessing the severity of patients with CAP receiving inpatient treatment [15]. However, when comparing the areas under the ROC curve between A-DROP and CURB-65, they detected a difference in the results. They reported that A-DROP had a greater area under the ROC curve than CURB-65 did; [15] meanwhile, we observed a greater area under the ROC curve for CURB-65. This may be explained by the difference in study populations—inpatients vs. outpatients.

In numerous previous studies, including international guidelines, PSI and CURB-65 have been documented to be helpful in assessing the severity of CAP [10, 18–22]. Man et al. found CURB-65 to be more suitable than PSI for use in the ED because of the simplicity of application and its ability to identify low‐risk patients [23]. Our study showed that A-DROP could be used to determine discharge readiness as well. Furthermore, because the area under the ROC curve for CURB-65 was greater than that for A-DROP, it could be used as a superior evaluation tool for discharging patients with CAP than A-DROP.

Almost all patients who revisited the hospital in our study were above the age of 65 years (72%). Older patients, including those with low-risk scores, should be particularly considered for admission to a short-term observation unit or ward, according to our findings.

Considering our hospital's clinical practice, 60% of non-low-risk patients were discharged without any CAP severity score determined using any of the available systems. This reflects the underutilization of such scoring systems, which are recommended by international guidelines, at our institution. Nevertheless, in a previous study [5] where patients were discharged based on either CURB-65 or CRB-65, the rate of revisit was very similar to that observed in our study—8.4% vs. 7.1%; similar findings were observed regarding the rate of discharge of non-low-risk patients—32.1% vs. 37.5%.

Many studies have shown that the severity scoring systems are of limited utility in deciding whether or not to admit patients with CAP. Clinical judgment should be added to clinical decision-making because other factors, such as the requirement of additional investigations, social support, and comorbidities, are to be considered. In addition, it is not uncommon for patients who are considered low risk to be managed in-hospital [24–26]. This is supported by our finding that some of the patients in the low-risk group died within 30 days after discharge.

The article "Comparison between the Severity Scoring Systems A-DROP and CURB-65 for Predicting Safe Discharge from the Emergency Department in Patients with Community-Acquired Pneumonia" was published in 2022. Journal: Emerg Med Int.

To the best of our knowledge, this is the first study to assess discharge readiness using these scoring systems in outpatients with CAP discharged from the ED; previous studies have included only inpatients. We hypothesized that in the low-risk score group, outpatient studies would provide a more accurate disease prognosis and superior clinical outcomes. However, our study has some limitations that are worth mentioning. First, it is a single-center study; thus, the results are difficult to generalize. Second, it was retrospective in nature, which could have resulted in selection bias because patients with incomplete data were excluded, and those who were discharged might have elected to visit other hospitals, which may have led to a lower rate of revisits and death.

## 5. Conclusions

There was no significant difference between the A-DROP and CURB-65 scoring systems in predicting the severity of condition in patients with CAP discharged from the ED. Prospective, multicenter studies are required to confirm these findings. Due to the high rate of revisit, older patients, even those with low-risk scores, should be particularly considered for admission to a short-term observation unit or ward.

## Figures and Tables

**Figure 1:** Study flow diagram showing patient selection. Abbreviations: CAP, community-acquired pneumonia; HAP, hospital-acquired pneumonia.

**Figure 2:** Receiver operating characteristic (ROC) curves for (—) A-DROP score and (- - -) CURB-65 score to predict the 30-day mortality rate in patients with community-acquired pneumonia. (....) Reference line.

**Figure 3:** Receiver operating characteristic (ROC) curves for (—) A-DROP score and (- - -) CURB-65 score to predict hospital revisit rate within 72 hours after discharge from the emergency department in patients with community-acquired pneumonia. (....) Reference line.

**Table 1:** Baseline characteristics and outcome measures in patients with community-acquired pneumonia.

Baseline characteristics and outcome measures	*N* = 408	30-day mortality, *N* = 6	Revisit within 72 hours, *N* = 29
**Baseline characteristics**			
Male, *N* (%)	214 (52.5)	3 (50.0)	17 (58.6)
Female, *N* (%)	194 (47.5)	3 (50.0)	12 (41.4)
Age (years)			
Mean (SD)	67.9 (17.9)	83.3 (12.5)	74.1 (15.1)
Median (IQR)	71 (58–81)	80 (78–94)	77 (63–84)
Age ≥65 years, *N* (%)	253 (62.0)	6 (100.0)	21 (72.4)
Male ≥70 years and female ≥75 years, *N* (%)	198 (48.5)	5 (83.3)	18 (62.1)
Comorbidities, *N* (%)			
Neoplastic disease	36 (10.9)	2 (33.3)	2 (6.9)
Chronic lung disease	82 (24.8)	3 (50.0)	4 (13.8)
Congestive heart failure	6 (1.8)	0 (0)	2 (6.9)
Chronic renal disease	40 (12.1)	1 (16.7)	7 (24.1)
Chronic liver disease	20 (6.1)	1 (16.7)	3 (10.3)
CNS disorder	82 (24.8)	3 (50.0)	10 (34.5)
Diabetes	88 (26.7)	1 (16.7)	8 (27.6)
Clinical parameters, *N* (%)			
Orientation disturbance (confusion)	10 (2.5)	0 (0)	2 (6.9)
Systolic blood pressure <90 mm Hg. or diastolic blood pressure ≤60 mm Hg	59 (14.5)	1 (16.7)	3 (10.3)
Pulse rate ≥125 bpm	14 (3.4)	0 (0)	1 (3.5)
Respiratory rate ≥30 BPM	103 (25.2)	5 (83.3)	14 (48.3)
SaO_2_ ≤ 90% (or PaO_2_ ≤ 60 mmHg)	28 (6.9)	1 (16.7)	6 (20.7)
Laboratory findings, *N* (%)			
BUN >20 mg/dL	97 (23.8)	4 (66.7)	10 (34.5)
BUN ≥21 mg/dL	89 (21.8)	4 (60.7)	9 (31.0)
Radiographical findings, *N* (%)			
Bilateral lung involvement ≥ two zones involved‡	26 (6.4)	0 (0)	4 (13.8)
Use of antibiotics within the previous 90 days, *n* (%)	43 (10.5)	0 (0)	2 (6.9)

*Outcome measures*			
Recovery, *N* (%)	379 (92.9)		
Revisit within 72 hours, *N* (%)	29 (7.1)		
Discharged	18 (62.1)		
Discharged then died within 30 days	1 (3.4)		
Admitted	10 (34.5)		
Admitted then died within 30 days	3 (10.4)		
30-day mortality, *N* (%)	6 (1.5)		

^‡^The lungs are divided into five zones: right and left upper, right and left lower, and right middle zones. Abbreviations: BPM, breaths per minute; bpm, beats per minute; BUN, blood urea nitrogen; CNS, central nervous system; IQR, interquartile range; SD, standard deviation.

The article "Comparison between the Severity Scoring Systems A-DROP and CURB-65 for Predicting Safe Discharge from the Emergency Department in Patients with Community-Acquired Pneumonia" was published in 2022. Journal: Emerg Med Int.

**Table 2:** Distribution of patients, 30-day mortality, and hospital revisit within 72 hours in each risk class assessed using the A-DROP and CURB-65 scoring systems.

Risk group	Number of patients *N* = 408	30-day mortality *N* = 6	Revisit within 72 hours *N* = 29
A-DROP score			
0	44.1 (180)	0.6 (1)	5.0 (9)
1	36.3 (148)	0.7 (1)	6.8 (10)
2	17.2 (70)	4.3 (3)	7.1 (5)
3	2.2 (9)	11.1 (1)	55.6 (5)
4	0.2 (1)	0 (0)	0 (0)
5	0 (0)	0 (0)	0 (0)
CURB-65 score			
0	26 (106)	0 (0)	3.8 (4)
1	37 (151)	0.7 (1)	5.3 (8)
2	25.5 (104)	1.9 (2)	9.6 (10)
3	10.0 (41)	4.9 (2)	14.6 (6)
4	1.5 (6)	16.7 (1)	16.7 (1)
5	0 (0)	0 (0)	0 (0)

Data are expressed as % (*N*).

**Table 3:** Distribution of the revisit group based on A-DROP and CURB-65 scores.

Clinical factors	Number of patients, *N* = 29
A-DROP score	
A: age (years) (male ≥70 and female ≥75)	18 (62.1)
D: dehydration (BUN ≥21 mg/dL)	9 (31.0)
R: respiratory failure (SaO_2_ ≤ 90% or PaO_2_ ≤ 60 mmHg)	6 (20.7)
O: orientation disruption (confusion)	2 (6.9)
P: low blood pressure (systolic blood pressure ≤90 mmHg)	0

*CURB-65 score*	
C: confusion	2 (6.9)
B: blood urine nitrogen >20 mg/dL	10 (34.5)
R: respiratory rate ≥30 breaths per minute	14 (48.3)
B: systolic blood pressure <90 mm Hg or diastolic ≤60 mmHg	3 (10.3)
A: age ≥65 years	21 (72.4)

BUN, blood urea nitrogen. Data are expressed as *N* (%).

The article "Comparison between the Severity Scoring Systems A-DROP and CURB-65 for Predicting Safe Discharge from the Emergency Department in Patients with Community-Acquired Pneumonia" was published in 2022. Journal: Emerg Med Int.

## Data Availability

The data used to support the findings of this study are available from the corresponding author upon request.
